The article "Histopathological, histochemical and biochemical postmortem changes in induced fatal hypothermia in rats" was published in 2021. Journal: Forensic Sci Res.

# Histopathological, histochemical and biochemical postmortem changes in induced fatal hypothermia in rats

**DOI:** 10.1080/20961790.2021.1886656

**Published:** 2021-06-14

**Authors:** Mahrous Abdelbasset Ibrahim, Sally Salem Mohammed, Hany Goda Tammam, Rehab Ibrahim Abdel-Karim, Medhat Mohammed Farag

**Affiliations:** a Forensic Medicine & Clinical Toxicology, College of Medicine, Jouf University, Sakakah, Saudi Arabia; b Forensic Medicine & Clinical Toxicology Department, Faculty of Medicine, Suez Canal University, Ismailia, Egypt; c Histology and Cell Biology Department, Faculty of Medicine, Suez Canal University, Ismailia, Egypt; d Forensic Medicine and Clinical Toxicology Department, Faculty of Medicine, Al-Azhar University, Cairo, Egypt; e Medical biochemistry Department, College of Medicine, Shaqra University, Shaqraa, Saudi Arabia; f Medical Biochemistry & Molecular Biology Department, Faculty of Medicine, Benha University, Benha, Egypt

**Keywords:** Forensic sciences, forensic medicine, legal medicine, autopsy, forensic pathology, histochemical, hypothermia

## Abstract

Reaching a postmortem diagnosis of hypothermia is challenging in forensic practice. Therefore, this study was conducted to detect the histopathological, histochemical and biochemical changes that occur in adult albino rats following exposure to induced fatal hypothermia. Twenty-four adult albino rats were divided into the negative control, moderate hypothermia, severe hypothermia and hypoxia groups. Rats in the control group were euthanized when those in the moderate hypothermic group died. Blood samples were collected *via* heart puncture, and the cerebrum, heart, suprarenal gland, kidney, liver and skeletal muscle were removed to investigate the biochemical, histochemical and histopathological changes. Postmortem assessment depicted significant changes in lipid peroxidation, represented by increased malondialdehyde levels in the studied organs of the rats in hypothermic and hypoxia groups. Histopathological examination of the rats’ organs revealed degeneration and necrosis in the hypothermia and hypoxia groups. Sections taken from the severe hypothermic rats revealed a loss of normal cardiac tissue architecture, necrotic changes in the pyramidal cells in the cerebral cortex, and massive necrosis, mainly in the tubules of the renal cortex and medulla. These findings suggest that histological changes might be used as biochemical markers for postmortem diagnosing of fatal hypothermia, particularly in severe hypothermic conditions.

**Key points**
- Death by hypothermia is a serious public health problem worldwide.
- Confirming a diagnosis and determining the cause of death in cases of hypothermia are among the most difficult practices in forensic medicine.
- Death by hypothermia might be associated with structural abnormalities in various organs.
- Studies using different tissue staining techniques will enable an overall illustration of the role of histopathological changes in body organs as indicators of hypothermia.

The article "Histopathological, histochemical and biochemical postmortem changes in induced fatal hypothermia in rats" was published in 2021. Journal: Forensic Sci Res.

## Introduction

A postmortem diagnosis of hypothermia remains difficult to ascertain despite the progress made in the field of forensic medicine in recent decades [1, 2]. Interest is currently growing in the postmortem diagnosis of hypothermia. Death by hypothermia is usually diagnosed based on circumstances and supported by a few non-specific findings at the autopsy. However, several cases have been diagnosed according to history and exclusion [3].

Hypothermia causes major dysfunction in the vital organs. Various pathological changes, including cutaneous [4,5], gastric [6], cardiac [7], renal [8] and pancreatic [9] changes, have been detected in hypothermia-induced fatalities. Frost erythema (reddish-brown discolouration of the skin over the elbows and knees) and Wischnewsky spots (acute gastric erosions) have been identified as classic signs of hypothermia [10], especially when both occur concomitantly. However, these classic morphological changes are insufficient for establishing an unequivo­cal diagnosis of death from hypothermia [11,12]. Furthermore, such changes are rarely detected in hypothermia-induced fatalities that occur while under the influence of ethanol because ethanol accelerates lowering the body temperature and hastens death [1].

Hypothermia is defined as a drop in core body temperature to ≤35°C. Below this temperature, the body loses more heat than it generates, causing a potentially fatal condition. Based on the core body temperature, the severity of hypothermia is categorized as either mild, moderate or severe. The core body temperature ranges from 32°C to 35°C under mild hypothermia and decreases to <28°C under severe hypothermia [12].

In legal medicine, hypothermia can be classified as either dry or wet hypothermia and can be further categorized into acute, subacute and chronic hypothermia. In acute hypothermia, the severe cold stress exceeds the body’s capacity to produce heat as a compensatory mechanism; hence, cooling occurs rapidly before the body energy stores are depleted. This often occurs after cold-water immersion. In subacute hypothermia, the body is exposed to less severe cold; hence, the body cools after complete depletion of energy stores. Chronic hypothermia results from many days of prolonged exposure to moderate cold and usually occurs in malnourished individuals suffering from chronic illnesses and older people living in destitute housing conditions. Young children are also more prone to developing hypothermia [2,13].

The article "Histopathological, histochemical and biochemical postmortem changes in induced fatal hypothermia in rats" was published in 2021. Journal: Forensic Sci Res.

Exposure to cold is a stressor that accelerates metabolic rates and helps generate reactive oxygen species (ROS). When ROS production exceeds the cellular antioxidative defence mechanisms, oxidative stress occurs [12,14].

Despite great scientific research efforts to identify more reliable diagnostic criteria for hypothermia-induced fatalities, significant advances in the field remain comparatively limited [15]. For several years, great effort has been devoted to studying the biochemical changes associated with hypothermia fatalities [10,14]. However, most previous studies did not account for the association between biochemical and pathological changes in the serum and tissues. Some stress biomarkers, such as heat shock protein 70 (Hsp70), were investigated as biomarkers of hypothermia in the renal tubular epithelial cells. Heat shock proteins are molecular chaperones expressed in the tissues of victims exposed to stress conditions. Although increased Hsp70 expression has been found in the kidneys in cases of hypothermia, it has not been strongly correlated with Wischnewsky spots. Furthermore, Hsp70 is non-specific for hypothermia and appears with other stress conditions such as ischaemia, burns and myocardial infarction [16].

Because little research has been conducted on this topic, the current study was conducted to detect the postmortem histopathological, histochemical and biochemical changes in the brain, heart, liver, kidneys, suprarenal gland and skeletal muscle of rats following experimental exposure to induced fatal hypothermia.

## Materials and methods

This study was performed in the Forensic Medicine & Clinical Toxicology Department in collaboration with the Histology & Cell Biology Department, Faculty of Medicine, Suez Canal University (SCU), Egypt. The Research Ethical Committee (REC), Faculty of Medicine, SCU (Research # 4230) approved the study, which complied with the Guide for Care and Use of Laboratory Animals published by the US National Institutes of Health (NIH Publication No. 85-23, revised 1996). The authors further attest that all efforts were made to minimize the number of animals used and the animals’ suffering.

Twenty-four 8–10-week-old albino rats weighing 200–220 g were used in the experiments. The rats were purchased from the National Centre of Research, Cairo, Egypt. They were allowed to acclimatise for 7 days before the experiment. The rats had free access to food and water and were maintained on a 12/12-h day/night cycle. The animals were randomly divided into four groups, with six rats per group [17] as follows.

The article "Histopathological, histochemical and biochemical postmortem changes in induced fatal hypothermia in rats" was published in 2021. Journal: Forensic Sci Res.

Rats in the negative control (NC) group were kept at room temperature ((23 ± 2)°C, as a normothermic condition) under standard housing at (45 ± 5)% humidity on a 12/12-h light/dark cycle.

Rats in the moderate hypothermia (MH) group were kept in cages in a refrigerator with the temperature set at 2°C–8°C (hypothermic conditions). The rats were left until they died (death occurred within 70–74 h in the refrigerator).

Rats in the severe hypothermia (SH) group were kept in cages in a deep freezer with the temperature set at −2 to 0°C (hypothermic conditions). The rats were left until they died (half died within the first 12 h; the other half died within the next 12 h).

Rats in the hypoxia (Hx) group were subjected to hypoxic insult as previously described [18]. These rats were added to the study to test whether the changes detected were specific to hypothermia or occurred under other stressful conditions such as hypoxia.

A rectal thermometer was used daily to measure the rats’ core body temperature to confirm that the core temperatures were 37°C (normothermic conditions) for the NC group, 28°C–32°C (moderate hypothermic conditions) for the MH group and ≤28°C (severe hypothermic conditions) for the SH group. The rats in the negative control group were euthanized when the rats in the MH group died.

### Histopathological and histochemical investigations

After the rats in the hypothermia and hypoxia groups died and those in the NC group were eutha­nized, the cerebrum, heart, suprarenal gland, kidneys, skeletal muscle and liver were obtained to study the histopathological and histochemical changes.

Half of the specimens were used for frozen tissue sections; the other half were fixed in formalin to use for paraffin-embedded tissue sections. The frozen sections were stained with oil red O to view the lipids. The paraffin blocks were sectioned at ∼4 µm and stained with haematoxylin and eosin (H&E) to view the general architecture of all collected organs. Additionally, special stains were performed for each organ according to the issue under study. Cerebral sections were stained with cresyl violet to demonstrate Nissl’s granules. The cardiac and skeletal muscle sections were stained with iron haematoxylin to show the cross-muscle striations. Renal sections were stained with periodic acid-Schiff (PAS) to visualize changes in the basal lamina, and hepatic sections were stained with Masson’s trichrome stain to view the connective tissue and collagen content.

### Biochemical investigations

1. Rats in the NC group were anaesthetized before euthanasia, and blood samples were collected *via* heart puncture. Blood samples were collected *via* direct heart puncture from rats in the MH, SH and Hx groups immediately after confirming death. Samples were left at room temperature until they clotted, then centrifuged at 3 000 rpm at 4°C for 15 min. Serum was separated from each sample and stored at −20°C as aliquots to be used for further analysis.

The article "Histopathological, histochemical and biochemical postmortem changes in induced fatal hypothermia in rats" was published in 2021. Journal: Forensic Sci Res.

The total protein, glucose, cholesterol and triglycerides in the serum were estimated colormetrically as previously described using kits from the Bio-diagnostic Company (Dokki, Egypt) [19–21].

Cardiac troponin I (cTnI) was measured as per the methods of Wu et al. [22]. Serum adrenocorticotropic hormone (ACTH) and cortisol levels were estimated according to the methods of Bańka et al. [23]. The serum adrenaline levels were measured according to Zhu et al. [24] and Ishikawa et al. [25]. The free fatty acids (FFAs) were measured according to Bańka et al. [26].

A calcium colorimetric assay kit was used to measure the calcium levels in the serum as per the methods of Leary et al [27]. at 575 nm and 0.4–100.0 mg/dL (0.1–25.0 mmol/L). The calmagite dye method was used to measure the serum magnesium levels according to the methods of Henry and AuBuchon [28]. To ensure the quality and accuracy of the measurements, two levels of the control sera were run with every batch.

1. The brain, heart, suprarenal gland, kidney, liver and skeletal muscle of six rats from each experimental group were rapidly excised. Part of each organ was washed with 0.9% NaCl solution, then blotted over a piece of filter paper and perfused with phosphate-buffered saline (50 mmol/L potassium phosphate pH 7.4) in an ice-containing medium. Subsequently, the tissues were homogenised in 5 mL cold buffer per g of tissue using a Dounce Tissue Grinder (Omni International, Kennesaw, GA, USA) and centrifuged at 4 000 rpm for 15 min at 4°C using a cooling centrifuge. The resulting supernatant was then transferred into Eppendorf tubes and kept at −80°C until used for various biochemical assays. Total antioxidant capacity (TAC) and lipid peroxidation products (malondialdehyde; MDA) were measured in the cardiac, renal, hepatic, suprarenal gland, brain and skeletal muscle tissues using kits from the Bio-diagnostic Company [29,30].

### Statistical analysis

Data were processed using SPSS software, version 23.0 for windows (IBM Corp., Armonk, NY, USA) and presented as the mean ± SD. One-way analysis of variance was used for comparisons, followed by Duncan’s multiple-range tests for *post hoc* analysis. *P* < 0.05 was considered statistically significant.

## Results

### Postmortem serum biomarkers in the hypothermic, Hx and NC groups

Table 1 summarizes the overall measurements, which represent the results of postmortem assessments of the serum biomarkers in the rats that died from induced hypothermia or hypoxia and the control group. Serum levels of the hormones cortisol, ACTH and adrenaline, the electrolytes Ca^2+^ and Mg^2+^, and cTnI were significantly increased in the SH group compared with those of the NC, MH and Hx groups (*P* < 0.05), with significant differences between the NC and MH and Hx groups (*P* < 0.05). Serum levels of FFAs (palmitic and stearic acid) were significantly decreased in the SH group compared with those of the NC, MH and Hx groups (*P* < 0.05); however, these levels were significantly increased in the MH and Hx groups compared with those of the NC group (*P* < 0.05).

The article "Histopathological, histochemical and biochemical postmortem changes in induced fatal hypothermia in rats" was published in 2021. Journal: Forensic Sci Res.

**Table 1.** Postmortem serum biomarkers in control rats and rats that died from induced hypothermia and hypoxia (*n* = 6/group).

Postmortem serum biomarkers	NC	MH	SH	Hx
Cortisol (ug/dL)	16.33 ± 1.03	28.67 ± 1.08^a^	34.67 ± 1.35^a^ ^b^ ^c^	25.33 ± 1.96^a^
ACTH (pg/mL)	11.81 ± 0.54	15.33 ± 1.09^a^	18.32 ± 0.63^a^ ^b^ ^c^	14.92 ± 0.88^a^
Adrenaline(ng/L)	36.03 ± 1.07	70.42 ± 4.59^a^	79.92 ± 2.85^a^ ^b^ ^c^	63.10 ± 3.22^a^
Troponin I (ng/mL)	0.005 ± 0.002	0.79 ± 0.09^a^	0.91 ± 0.04^a^ ^b^ ^c^	0.66 ± 0.06^a^
Calcium (mg)	12.35 ± 1.24	16.32±0.93^a^	20.05 ± 1.02^a^ ^b^ ^c^	14.75 ± 0.52^a^
Magnesium (mg)	4.70 ± 0.76	8.10 ± 0.64^a^	11.07 ± 0.78^a^ ^b^ ^c^	7.72 ± 0.38^a^
Palmitic acid (µEq/L)	571.17 ± 22.39	704.17 ± 21.41^a^	459.67 ± 23.51^a^ ^b^ ^c^	686.67 ± 14.73^a^
Stearic acid (µEq/L)	55.33 ± 2.66	66.83 ± 2.64^a^	43.72 ± 1.69^a^ ^b^ ^c^	64.17 ± 2.04^a^
Glucose (mg/dL)	115.67 ± 5.50	69.66 ± 3.67^a^	79.00 ± 4.73^a^ ^b^ ^c^	66.67 ± 1.97^a^
Triglycerides (mg/dL)	61.67 ± 3.27	82.50 ± 5.99^a^	86.17 ± 5.04^a^	78.50 ± 3.94^a^
Cholesterol (mg/dL)	86.17 ± 2.48	72.83 ± 2.32^a^	73.16 ± 3.31^a^	75.67 ± 2.66^a^
Total protein (g/dL)	12.28 ± 0.38	11.95 ± 0.63	12.02 ± 0.26	11.78 ± 0.72

Data are the mean ± SD. Significant at *P* < 0.05.

NC: negative control group; MH: moderate hypothermic group; SH: severe hypothermic group; Hx: hypoxia group; ACTH: adrenocorticotropic hormone.

a Compared with the NC group.

b Compared with the MH group.

c Compared with the Hx group.

Serum glucose levels were significantly decreased in the MH, SH and Hx rats compared with those of the NC group (*P* < 0.05). Serum triglycerides level were significantly increased in the MH, SH and Hx rats compared with those of the NC group (*P* < 0.05). Serum cholesterol levels were significantly reduced in the MH, SH and Hx rats compared with those of the NC rats (*P* < 0.05). However, the triglyceride and cholesterol levels did not differ between the MH, SH and Hx groups (*P* > 0.05). Serum total proteins differed only insignificantly between the four groups, and all investigated parameters differed only insignificantly between the MH and Hx groups.

The article "Histopathological, histochemical and biochemical postmortem changes in induced fatal hypothermia in rats" was published in 2021. Journal: Forensic Sci Res.

### Postmortem tissue lipid peroxidation and TAC

Postmortem assessment of the tissue lipid peroxidation in the rats that died from induced hypothermia and hypoxia showed significant changes in the lipid peroxides as represented by increased MDA levels in the brain, heart, liver, kidney, suprarenal gland and skeletal muscle tissues among all four groups (*P* < 0.05; Table 2). Lipid peroxide levels were significantly increased in the MH, SH and Hx groups compared with those of the NC group. MDA levels were significantly increased in the SH group compared with those of the MH and Hx groups (*P* < 0.05) in all investigated organs except the kidneys. MDA levels did not significantly differ between the MH and Hx groups.

**Table 2.** Postmortem levels of tissue lipid peroxidation and total antioxidants in control rats and rats that died from induced hypothermia and hypoxia (*n* = 6/group).

Tissue	NC	MH	SH	Hx
*MDA (nmol/g)*				
Brain	9.77 ± 0.34	17.22 ± 1.45^a^	25.08 ± 2.58^a^ ^b^ ^c^	15.38 ± 0.90^a^
Heart	11.30 ± 1.45	18.50 ± 1.76^a^	28.30 ± 2.89^a^ ^b^ ^c^	16.47 ± 0.37^a^
Liver	14.20 ± 2.20	22.50 ± 2.34^a^	26.20± 3.23^a^ ^b^ ^c^	20.17 ± 1.33^a^
Kidney	12.80 ± 1.78	21.40 ± 2.12^a^	23.60 ± 3.18^a^	19.17 ± 1.47^a^
Suprarenal gland	8.40 ± 0.97	16.40 ± 1.65^a^	24.70 ± 2.68^a^ ^b^ ^c^	14.57 ± 1.33^a^
Skeletal muscle	11.55 ± 1.30	18.03 ± 0.53^a^	26.98 ± 1.09^a^ ^b^ ^c^	14.65 ± 0.75^a^
*TAC (µmol/g)*				
Brain	0.538 ± 0.045	0.265 ± 0.037^a^ ^c^	0.232 ± 0.054^a^ ^c^	0.397 ± 0.039^a^
Heart	0.632 ± 0.067	0.324 ± 0.076^a^ ^c^	0.289 ± 0.014^a^ ^c^	0.446 ± 0.024^a^
Liver	0.768 ± 0.052	0.564 ± 0.044^a^ ^c^	0.345 ± 0.058^a^ ^b^ ^c^	0.620 ± 0.041^a^
Kidney	0.711 ± 0.065	0.544 ± 0.076^a^ ^c^	0.312 ± 0.036^a^ ^b^ ^c^	0.593 ± 0.015^a^
Suprarenal gland	0.522 ± 0.038	0.253 ± 0.012^a^ ^c^	0.233 ± 0.024^a^ ^c^	0.312 ± 0.017^a^
Skeletal muscle	0.583 ± 0.063	0.255 ± 0.027^a^ ^c^	0.225 ± 0.026^a^ ^c^	0.335 ± 0.075^a^

Data are the mean ± SD. Significant at *P* < 0.05.

NC: negative control group; MH: moderate hypothermic group; SH: severe hypothermic group; Hx: hypoxia group; MDA: malondialdehyde; TAC: total antioxidant capacity.

a Compared with the NC group.

b Compared with the MH group.

c Compared with the Hx group.

The TAC in all organ tissues was significantly reduced in the MH, SH and Hx groups compared with that of the NC group, with no significant differences between the MH and SH groups except in the liver and kidneys. The TAC in the liver and kidneys was decreased significantly in the SH group compared with that of the MH group (*P* < 0.05). Furthermore, TAC levels were significantly decreased in the MH and SH groups compared with those of the Hx group.

The article "Histopathological, histochemical and biochemical postmortem changes in induced fatal hypothermia in rats" was published in 2021. Journal: Forensic Sci Res.

### Histopathological and histochemical results

Five fields from three sections per animal were examined.

#### Histopathological and histochemical changes in the cerebral cortex

H&E-stained sections of the NC group revealed normal architecture of the cerebral cortex with normal pyramidal cells, basophilic cytoplasm and large rounded central nuclei with prominent nucleoli, longitudinally directed nerve fibres between the cells and normal clear blood capillaries (Figure 1A). H&E-stained sections from the MH and SH rats revealed necrotic pyramidal cells. These cells were more rounded and had more acidophilic cytoplasm, absent nucleoli with karyolytic nuclei and fragmented chromatin in the SH group. Some areas had a complete loss of cells and decreased longitudinal intercellular nerve fibres compared with those of the control group. Increased acidophilia with engorged blood capillaries and tissue detachment were detected, especially in the SH group (Figure 1B and C). Hypoxic H&E-stained brain sections contained many areas with congested blood capillaries, haemorrhaging and oedema, with pyknotic cells (Figure 1D). Cresyl violet-stained sections of the NC group tissues showed deep purple staining in the cytoplasm of the pyramidal cells and the beginning of the axons (Nissl’s granules; Figure 1E). The pyramidal cell cytoplasm in the MH and SH groups stained a lighter purple than that of the NC group owing to the loss of Nissl’s granules (Figure 1F and G). The hypoxic brain tissue contained violet-stained cytoplasm (Nissl’s granules) like that of the NC group (Figure 1H).

**Figure 1.** Photomicrograph of transverse section in the rat brain stained with H&E (×60) (A–D) and Cresyl violet (×100) stains (E–H). (A) Negative control (NC) group showing normal pyramidal cells (arrow heads) with basophilic cytoplasm, rounded nucleus and prominent nucleolus. Clear blood capillaries (arrows) with normal fibrous appearance. (B) Moderate hypothermia (MH) group showing necrotic pyramidal cells with acidophilic cytoplasm and karyolytic nuclei (arrow heads), other areas show loss of cells (*). Engorgement of blood capillaries (arrows) with decrease in the longitudinal nerve fibre appearance. (C) Severe hypothermia (SH) group showing necrotic pyramidal cells with acidophilic cytoplasm. Some show karyolytic nuclei (arrow heads), others show fragmentation of their chromatin (arrow) with severe detachment in the tissue (*). (D) Hypoxia (Hx) brain shows areas with red blood cells (RBCs) and edema in the brain tissue (arrow heads) with pyknotic nuclei (arrow). (E) NC group showing deep purple staining of the cytoplasm around the nuclei and in the axon beginning (arrows). (F) MH group showing light purple staining of the cytoplasm (arrows). (G) SH group also has light purple staining of the cytoplasm (arrows). (H) Hx group shows pyramidal cells with violet-stained cytoplasm indicating Nissil’s granules like the NC (arrows).

The article "Histopathological, histochemical and biochemical postmortem changes in induced fatal hypothermia in rats" was published in 2021. Journal: Forensic Sci Res.

#### Histopathological and histochemical changes in the cardiac muscle

H&E- and iron haematoxylin-stained sections from the NC group revealed normal cardiomyocytes and cross-striations of their cytoplasm. The cardiomyocytes were separated by minimal connective tissue (Figure 2A and E). H&E-stained sections from the MH and SH groups revealed a loss of the normal cardiac tissue architecture with necrotic changes and haemorrhaging (Figure 2B and C). Iron haematoxylin-stained sections revealed a complete loss of the cross-striations in the cytoplasm of the cardiomyocytes, with severe haemorrhaging between cells (Figure 2F and G). In contrast to the hypothermic groups, the cardiac muscles of the Hx group had normal cytoplasm, and their nuclei had normal cross-striations, but these were worn out and separated by haemorrhaging (Figure 2D and H). Oil red O-stained frozen sections from all four groups revealed no lipid granules (Figure 2I).

**Figure 2.** Photomicrograph of transverse section in the rat heart stained with H&E (A–D), iron haematoxylin (E–H) and red oil stains (I) (×40). (A) Negative control (NC) group showing normal branched anastomosed cardiomyocytes with central oval vesicular nucleus. The cells are separated with little amount of connective tissue (arrows). (B) Moderate hypothermia (MH) group showing loss of arrangement of the cardiomyocytes with destruction of the cells and pyknotic nuclei (arrows). Wide spaces between the cardiomyocytes with haemorrhage (↔). (C) Severe hypothermia (SH) group showing destruction of the cells, pyknotic (arrows) and karyolytic (arrow heads) nuclei. Severe haemorhage between cardiomyocytes (*). (D) Hypoxia (Hx) group cardiomyocytes has normal cytoplasm and nuclei, but spaced and worn out with haemorrhage and edema (arrows). (E) NC group showing normal cross-striations of cardiomyocytes cytoplasm. (F) MH group showing complete loss of the cytoplasmic cross-striations of the cardiomyocytes (arrows) and severe haemorrhage between the cells (↔). (G) SH group showing loss of the cross-striations (arrow) and wide spaces with haemorrhage. (H) Cardiac muscle fibres still show cytoplasmic striations in spite of hypoxia (arrows). (I) Photomicrographs from the four groups show negative reaction for red oil stain.

The article "Histopathological, histochemical and biochemical postmortem changes in induced fatal hypothermia in rats" was published in 2021. Journal: Forensic Sci Res.

#### Histopathological and histochemical changes in the suprarenal gland

H&E-stained sections from the NC group revealed normal adrenal cortices and medullas in fibrous connective tissue capsules (Figure 3A). Oil red O-stained frozen tissue sections revealed no lipids in the capsule, zona reticularis or adrenal medulla; however, red-stained lipid granules were obvious in the zona glomerulosa and to a lesser extent in the zona fasciculata (Figure 3E).

**Figure 3.** Photomicrograph of longitudinal section in the rat suprarenal gland (cortex & medulla) stained with H&E (×40) (A–D) and red oil (×10) (E–H). (A) NC group showing capsule (C) zona glomerulosa (G) has small normal columnar acidophilic cells (arrow) around blood capillary with dark nuclei. Zona fasiculata (F) shows columns of foamy acidophilic spongiocytes around blood capillaries (arrow heads) with vesicular nuclei. Zona reticularis (R) shows anastomosing cords of acidophilic polyhedral cells with vesicular nuclei and lipofuscin pigments (triangular arrowhead). Medulla (M) shows wider blood capillaries (*) surrounded by clusters of chromaffin cells with vesicular nuclei. (B) Moderate hypothermia (MH) group showing similar picture to the NC group except for the congestion in medullary vessels (*). (C) Severe hypothermia (SH) group showing similar result to the MH group with more congestion in blood vessels between the cells of all layers (arrows) and in medulla (BL.V.). (D) Hypoxia (Hx) group showing suprarenal gland shows shrunken pyknotic cells of zona glomeruloza (G), wide spacing between all cells and empty sinusoids and capillaries from blood (*). (E) NC group showing the red oil stained lipid granules in the different layers of the adrenal gland. Negative reaction in the capsule (C) zona reticularis (R) and adrenal medulla (M). Red-stained granules in the cells of zona glomerulosa (G) and fasiculata (F) MH group showing increase in the red oil stained lipid granules in the suprarenal cortex (arrows), compared to the NC group. (G) SH group showing massive increase in the red oil stained granules in glomerulosa (G) and fasiculata (F) negative reaction in the C, R and M. (H) Hx group showing suprarenal cortex with red-stained lipids in zona fasiculata (F), like NC group.

H&E-stained sections from the MH group revealed similar results to those of the control group but with congested blood vessels in the suprarenal cortex and medulla (Figure 3B). Oil red O-stained sections revealed statistically significant increases in the lipid content of the suprarenal cortical cells compared with that of the NC group (Figures 3F and 4A).

H&E-stained sections from the SH group revealed severe congestion in the cortical and medullary vessels compared with those of the MH group (Figure 3C). Oil red O-stained sections revealed statistically significant increases in the lipid granule content in the cells of the zona glomerulosa and fasciculata compared with those of the other groups but no increases in the reticularis or adrenal medulla (Figures 3G and 4A).

The article "Histopathological, histochemical and biochemical postmortem changes in induced fatal hypothermia in rats" was published in 2021. Journal: Forensic Sci Res.

H&E- and oil red O-stained sections from the Hx group revealed comparable results to those of the control group except for the shrunken cells and blood loss in the capillaries (Figures 3D, H and 4A).

#### Histopathological and histochemical changes in the kidneys

H&E- and PAS-stained sections from the NC group revealed normal renal cortex, medulla and basal laminar structures (Figure 5A and E). Oil red O-stained sections revealed no lipids in either the renal cortex or medulla (Figure 6A).

**Figure 5.** Photomicrograph of transverse section in the rat kidney stained with H&E (A–D), PAS (E–H) (×40) stains. (A) Negative control (NC) group showing normal renal cortex and medulla. The cortex shows normal glomeruli (G) surrounded by patent urinary space (US), proximal convoluted tubules (PT) have narrow lumen and lined with large acidophilic cells that have rounded vesicular nuclei, also it shows distal convoluted tubules (DT) with wide lumen lined with cubical light acidophilic cells. Normally renal medullary tubules (MT). (B) Moderate hypothermia (MH) group showing necrosis in the cells lining medullary tubules, karyolysis (arrow head) and pyknosis in their nuclei (arrows) or loss of cells (**). Congestion in the blood capillaries (BC) of the cortex and medulla. Necrosis in the cortex also with increased acidophilia, pyknotic nuclei (arrow), complete loss of the nuclei (arrow head), obliteration of the renal tubules lumen and disappearance of the urinary space around the glomeruli (G). (C) Severe hypothermia (SH) group showing massive necrosis and loss of normal archeticture (*) and congested blood vessels (arrows). Complete necrosis of renal corpuscles (G). (D) Hypoxia (Hx) group kidney has complete lysis and loss of DCT cells, necrosis of PCT cells and shedding into lumen. Collapse of glomeruli (G), pyknosis and loss of cells lining the collecting ducts in medulla (M). (E) NC group showing regular thin basal lamina (arrows) surrounding the medullary tubules, the renal corpuscle (G), DT and PT. Cells of PT shows apical brush border (*). (F) MH group showing irregular basal lamina (arrows) in the renal cortex and medulla, or completely lost around the tubules (arrow heads). (G) SH group showing irregular basal lamina (arrows) and loss in other areas (*). (H) Hx group shows loss of basement membranes around renal tubules and glomeruli (arrows).

The article "Histopathological, histochemical and biochemical postmortem changes in induced fatal hypothermia in rats" was published in 2021. Journal: Forensic Sci Res.

**Figure 6.** Photomicrograph of transverse section in the rat kidney stained with red oil stain (×40). (A) Negative control (NC) group showing negative lipid content in the cortex and medulla. (B) Moderate hypothermia (MH) group showing positive lipid content in the cells lining the renal tubules. (C) Severe hypothermia (SH) group showing positive lipid content in the cells lining the medullary tubules. (D) Hypoxia (Hx) group showing negative lipid content in the cortex and medulla (red oil stain).

H&E-stained sections from both hypothermic groups revealed a complete loss of normal renal architecture. Necrosis occurred in all cells in the renal cortex and medulla, with congested blood capillaries (Figure 5B and C). PAS-stained sections revealed areas with an irregular or complete loss of basal lamina (Figure 5F and G). Oil red O-stained sections revealed increased lipid content in the cells lining the medullary tubules compared with that of the NC group (Figure 6B and C).

H&E- and PAS-stained sections in the Hx group revealed massive necrosis of the kidneys, with shedding of the cells lining the renal tubules and a loss of the basal laminae (Figure 5D and H). Oil red O staining revealed a negative reaction (Figure 6D).

#### Histopathological and histochemical changes in the liver

H&E-stained sections from the NC group revealed normal hepatic architecture (Figure 7A). Masson trichrome-stained sections revealed normal collagen fibre amounts around the central vein and portal tract with normally arranged hepatic cords separated by blood sinusoids (Figure 7E).

**Figure 7.** Photomicrograph of transverse section in the rat liver stained with H&E (A–D) and Masson’s trichrome (E–H) stains (×40). (A) Negative control (NC) has normal liver section with its central vein (CV), blood sinusoids (BL.S.) and cells arranged radially toward the CV. Hepatocytes are arranged in anastomosing cords with deep acidophilic cytoplasm and vesicular rounded nuclei with obvious nucleoli (arrow heads). (B) Moderate hypothermia (MH) group showing severe damage of the hepatocytes and engorgment of the CV and BL.S. with blood thinning out the hepatic cords. The hepatocytes have many cytoplasmic vacuolations (arrow heads) and karyolytic nuclei in some cells (arrows). (C) Severe hypothermia (SH) group showing also congestion of the CV and BL.S. Many hepatocytes show karyolytic nuclei (arrow heads) with heamosiderin deposits. (D) Hypoxia (Hx) liver shows congition of the portal vein and sinusoids (arrow heads), vacuolations of hepatocytes with karyolysis and loss of nuclei (arrows). (E) NC group showing normal collagen fibre amount around the central vein CV (arrows). Normally arranged hepatic cords spaced with blood sinusoids (arrow heads). (F) MH group showing dilated congested CV and blood sinusoids (arrows) with thinning of the hepatic cords. Little collagen fibers around CV. (G) SH group showing widely spaced blood sinusoids with red blood cells (arrows). Preservation of the collagen around the CV. (H) hypoxic liver shows normal content and distribution of greenish collagen fibers (arrow). (I) Micrograph from frozen liver showing negative lipid content in the four groups.

The article "Histopathological, histochemical and biochemical postmortem changes in induced fatal hypothermia in rats" was published in 2021. Journal: Forensic Sci Res.

H&E-stained sections from the MH group revealed liver damage with a loss of normal architecture (Figure 7B). Masson trichrome-stained sections revealed significantly decreased collagen content and thinning of the hepatic cords compared with that of the NC group (Figures 7F and 4B).

**Figure 8.** Photomicrograph of cross and longitudinal sections from the rat skeletal muscle stained with H&E (×40) (A–D) and iron hematoxyllin (×60) (E–H) stains. (A) Negative control (NC) group skeletal muscle fibres have cross-sections with multinucleated peripheral nuclei (arrow head) and rough cytoplasm (arrows). (B) Moderate hypothermia (MH) group showing normal cross-sections (arrows) except few cells show smooth light cytoplasm (arrow heads). (C) Severe hypothermia (SH) group showing that all sections have very light smooth cytoplasm (arrow). (D) Hypoxia (Hx) group showing normal appearance compared to NC group, but wide spacing between the muscle fibres. Iron haematoxylin section (E) longitudinal sections from NC group have normal cross-striations. (F) MH group showing normal cross-striations but with thinning out of the cells compared to control group. (G) SH group showing faint striations. (H) Hx group showing normal cross-striations of the cells but with wide spacing inbetween. (I) Red oil stained sections from the four groups revealed negative fat content.

H&E-stained sections of the SH group also revealed congestion of the liver tissue, with many hemosiderin deposits (Figure 7C). Masson trichrome-stained sections revealed dilatation of the hepatic sinusoids compared with those of the NC group, but unlike that in the MH group, the collagen content was preserved as in the NC group (Figures 7G and 4B).

H&E-stained sections of the Hx group livers revealed results similar to those of the MH group, but with normal collagen content compared with that of the NC group (Figures 7D, H and 4B). Frozen sections from all four groups revealed no lipids (Figure 7I).

#### Histopathological and histochemical changes in the skeletal muscle

The H&E- and iron haematoxylin-stained sections from the NC group appeared normal, with multinucleated muscle cells and deep acidophilic rough cytoplasm with obvious regular striations in the iron-stained longitudinal sections (Figure 8A and E).

The article "Histopathological, histochemical and biochemical postmortem changes in induced fatal hypothermia in rats" was published in 2021. Journal: Forensic Sci Res.

**Figure 4.** The mean ±SD of the colour area percentage of the (A) red oil stained fat in the suprarenal gland cortex and (B) the colour area percentage of the green stained collagen in the liver. a, Significant difference compared to Negative control (NC); b, Significant difference compared to moderate hypothermia (MH); c, Significant difference compared to hypoxia (Hx).

The H&E-stained cross-sections from the MH group showed skeletal muscle fibres similar to those of the NC group. The iron-stained skeletal fibres had normal cross-striations, but the fibres looked smaller than those of the NC group (Figure 8B and F).

All H&E-stained sections from the SH group showed light acidophilic smooth skeletal fibres, with weak cross-striations on the iron-stained sections (Figure 8C and G).

The H&E- and iron haematoxylin-stained sections from the Hx group had comparable results to those of the NC group, except for wide spacing between the skeletal fibres (Figure 8D and H). All four groups lacked lipids in the frozen tissue sections when stained with oil red O (Figure 8I).

## Discussion

A postmortem diagnosis of hypothermia is difficult to ascertain because it depends heavily on the exclusion of other possible causes of death [2]. Thus, the current study was conducted to establish the diagnostic criteria of induced fatal hypothermia in rats based on biochemical and histopathological parame­ters of different organs.

Cognitive, emotional and biological factors are associated with stress as a complex condition. Many changes in the human body are associated with persistent stress in the form of short- and long-term disability. Additionally, exposure to stress activates the central nervous system’s defence mechanisms [31]. Because hypoxia is a stressor, altered stress responses, such as increased ACTH and glucocorticoids along with their consequent metabolic changes, can be expected [32].

In the present study, the ACTH, cortisol and adrenaline levels increased significantly in the hypothermic groups compared with those of the NC group. These findings are consistent with previous animal studies [17,33] and postmortem human studies [34]. However, Palmiere et al. [35] reported normal ACTH levels, assuming that these levels might be initially increased in response to cold exposure, then depressed in delayed stages. Exposure to stress, including cold, stimulates the hypothalamic–pituitary–adrenal axis and causes sympathetic overstimulation [25], which explains the elevated levels of these markers. Furthermore, the increased cortisol levels might be related to reduced hepatic clearance or stress-induced increased secretion [35].

The article "Histopathological, histochemical and biochemical postmortem changes in induced fatal hypothermia in rats" was published in 2021. Journal: Forensic Sci Res.

The previously mentioned markers are released in high levels during other stress-related causes of death; hence, we cannot rely on them as sole diagnostic criteria for hypothermia-induced fatalities. Furthermore, various factors, including postmortem interval, sampling techniques, sample preservation, endocrine disorders, metabolic dysfunctions and blood ethanol levels affect the levels of these mar­kers [12]. Immunohistochemical staining for ACTH was positive and showed similar expression patterns in autopsy cases for both the hypothermia and control groups [10]. cTnI is a highly sensitive and specific marker indicative of myocardial cell damage [36,37]. Consistent with Elshama et al. [17], we found significantly increased cTnI levels in the hypothermic groups compared with those of the NC group, and these levels were directly proportional to the intensity of the cold exposure. Hypothermia-induced cardiac injury was attributed to vasoconstriction and increased blood viscosity with consequent hypercoagulability [38]. This injury led to circulatory failure, ventricular arrhythmias and ischaemic-like echocardiographic changes associated with the elevated cTnI [39]. Conversely, Palmiere et al. [35] observed normal or mildly elevated serum cTnI levels in hypothermia-related fatalities as well as in some control subjects, suggesting myocardial hypoxia without severe myocardial damage in both hypothermia and control fatalities. A previous study found significantly increased cTnI levels in the blood plasma of rats exposed to severe hypobaric hypoxia for 3 h compared with those of the control group, thus indicating myocardial injury [40].

Consistent with the findings of Elshama et al. [17], serum calcium and magnesium were significantly increased in the present study. During mild hypothermia, renal blood flow increases owing to peripheral vasoconstriction, followed by decreased distal tubular reabsorption of water, and finally fai­lure to reabsorb water (cold diuresis) and increased electrolyte loss in the urine. However, during MH, renal blood flow decreases due to reduced cardiac output, leading to a reduced glomerular filtration rate. As the temperature progressively decreases, renal tubular secretion of hydrogen ions decreases, thus contributing to acidosis and electrolyte disturbances [41].

Postmortem human studies have reported lower calcium and magnesium levels in the pericardial fluid from hypothermic fatalities compared with those of the controls [35] and lower magnesium and higher calcium compared with those from other fatalities [42]. Jakubeniene et al. [43] found no significant changes in the calcium content of postmortem tissue.

The article "Histopathological, histochemical and biochemical postmortem changes in induced fatal hypothermia in rats" was published in 2021. Journal: Forensic Sci Res.

In the current study, both the hypothermia groups exhibited significantly lower glucose levels than those of the control group. Coe et al. [44] detected elevated glucose levels in some, but not all, hypothermia-related fatalities. Sympathetic overstimulation in response to stress, including cold exposure, initiates various metabolic changes. Catecholamine release induces gluconeogenesis and glycogenolysis, elevating glucose levels. Furthermore, increased corticosteroids inhibit insulin release and decrease insulin tissue uptake leading to initial hyperglycaemia [41]. The hypoglycaemia in both hypothermic groups in our study may have occurred as a result of shivering and depletion of glycogen stores to increase heat production, particularly when the duration of the hypothermia exposure increased [41]. In rats and small animals, non-shivering thermogenesis occurs in brown adipose tissue (BAT) [45]. During exposure to cold, BAT takes up excess glucose to generate heat, thus contributing to hypoglycaemia [46].

The significantly increased glucose levels in the SH group compared with those of the MH group may have been due to the shorter survival duration and lower metabolic rate and hence lower glucose consumption. Additionally, during SH, the glome­rular filtration rate decreases owing to decreased renal blood flow, which leads to decreased glucose clearance by the kidneys [41].

The current study revealed higher palmitic and stearic acid levels in the MH group than in the SH and NC groups. Lipids are considered impor­tant fuel sources [47]. Fat catabolism and triglyce­ride hydrolysis increase in response to cold exposure owing to the effects of stress hormones (i.e. glucagon, adrenaline, noradrenaline, cortisol and growth hormone), eventually elevating the FFA levels [14,48,49]. Glycolysis and β-oxidation of fatty acids in the BAT play major roles in heat production [46]. FFA levels were significantly lower in the SH group than those in the NC and MH groups. These findings were consistent with those of other postmortem animal studies [17], possibly owing to the short survival period in this group with the consequent inability to accumulate large amounts of FFAs in the blood or because of the decreased lipolysis [17].

In the current work, the hypothermia groups exhibited significantly increased triglycerides, decreased cholesterol and non-significant changes in total proteins levels compared with those of the NC group. This partially agreed with the results of Al-Ayadhi et al. [50], who detected decreased cholesterol and protein levels and elevated triglyceride levels in rats exposed to −10°C for 3 h. Devi and Manjula [51] observed increased total cholesterol and triglyceride levels during intermittent cold exposure (5°C and 10°C for 2 h/day). Those levels correlated positively with oxidative stress in the hippocampus. A previous study [52] reported that exposure to cold at 8°C for 2 days decreased protein, cholesterol and triglyceride levels in Sprague-Dawley rats.

The article "Histopathological, histochemical and biochemical postmortem changes in induced fatal hypothermia in rats" was published in 2021. Journal: Forensic Sci Res.

Cold stress initially increases the thyroid-stimulating hormone (TSH) and consequently raises thyroxin levels, which lowers total cholesterol levels [53]. With advanced hypothermia, TSH levels are suppressed owing to abnormal metabolism [53]. Differences in results between studies may be attributed to variability in the animal species and different experimental conditions [50]. The non-significant changes in serum total protein levels in the hypothermia groups compared with those of the NC group were attributed to the sparing effects of lipids and carbohydrates, which are considered the primary fuel for energy production, followed by proteins. Therefore, the intensity and duration of the cold exposure, as well as the duration of survival before death, are important factors affecting protein catabolism and hence total protein levels in the blood [54,55].

The present study revealed increased oxidative stress represented by significantly increased lipid peroxidation (MDA) levels and decreased TAC in the studied organs of the hypothermic groups compared with those of the NC group. Mammals increase energy production in response to cold exposure *via* two mechanisms: shivering (in the skeletal muscles) and non-shivering thermogenesis (in the BAT) [56]. Exposure to cold increases the metabolic rate, during which both oxygen consumption and ROS formation increase in different organs [57–59]. Consequently, ROS increase the oxidative damage to DNA, lipids and proteins and decrease the antioxidant activity in different tissues, including liver cells, hearts and rat brains [51,56,60]. This is attributed to the increased release of stress-induced corticosterone. Furthermore, lipid peroxidation products and hydrogen peroxide (H_2_O_2_) were found to be directly proportional to increased cold intensity [51]. Zhou et al. [60] observed that the MDA levels and TAC varied among tissues in response to cold exposure, which was also observed in the present study. Furthermore, these authors assumed that the response to cold exposure might vary with the duration of the exposure, the species exposed and the types of tissues studied.

A leftward shift of the oxygen dissociation curve, with an inability of haemoglobin to release oxygen to the cells, has been recorded as a pathophysiological mechanism in hypothermia. This hypoxia is associated with subsequent disturbances in fatty-acid metabolism and increased oxidative stress and eventually leads to degeneration and lipid accumulation in various tissues and organs in hypothermia-related fatalities [8,41]. Additionally, increased blood viscosity and elevated levels of cold agglutinins cause occlusion of the small blood vessels in tissues and organs, leading to micro-infarct formation and tissue degeneration [2].

The article "Histopathological, histochemical and biochemical postmortem changes in induced fatal hypothermia in rats" was published in 2021. Journal: Forensic Sci Res.

In the current work, histopathological examination of the cardiac muscles revealed loss of striations, haemorrhaging and necrosis. These changes explained the elevated cTnI levels in the rats and are consistent with the results of other animal studies [17] and of postmortem tissues from hypothermia-related fatali­ties [5]. Studies have reported that fatty degeneration of cardiac myocytes does not have the same sensitivity as that of renal fatty degeneration. Pathological changes in the cardiac tissue were attributed to hypoxia and the inability of haemoglobin to release oxygen to the tissues [7].

The present study revealed degenerative changes in the brain and engorged blood capillaries, which supports the findings of Elshama et al. [17]. These changes occurred in response to decreased cerebral blood flow and cerebral metabolic rates during hypothermia [61] and to the neurotoxic effects produced by excess free radicals and the metabolites of catecholamines [62]. Although antioxidant enzyme levels are initially elevated in brains exposed to mild and moderate hypothermia, they eventually become exhausted after prolonged exposure or during exposure to severe hypothermic conditions [60,63,64] as was shown in the current work. Neuroinflammatory changes, apoptosis of the hippocampal neurons, microglial activation and disrupted neurotransmitter release have been detected in response to hypothermia [65].

Consistent with other studies, we detected lipid granule accumulation and blood vessel congestion in the suprarenal glands in the hypothermia groups [2,8,17]. Furthermore, the degenerative changes in the renal and hepatic tissues in the present study were consistent with those reported in previous studies [5,8,12]. Fatty renal tubular degeneration was reported to have the most important diagnostic value in hypothermia-associated fatalities [8].

Our histological examination of rat skeletal muscles revealed nearly normal appearances, with some cells exhibiting smooth light cytoplasm. Exposure to cold stimulates oxidative stress; however, various tissues respond differently, which affects their survival and hence their damage in response to cold [56,60]. According to Zhou et al. [60], the uncoupling protein, UCP_3_, is upregulated in skeletal muscle mitochondria, leading to attenuation of the ROS production in these muscles and hence to less damage due to cold exposure. Their findings support the “uncoupling to survive” theory. Cold exposure for a short duration (24 h) in rats promoted protein degradation and decreased protein synthesis in skeletal muscles. However, noticeable atrophic changes were detected in the skeletal muscles after cold exposure for longer durations [63].

The article "Histopathological, histochemical and biochemical postmortem changes in induced fatal hypothermia in rats" was published in 2021. Journal: Forensic Sci Res.

Hypoxia stimulates anaerobic metabolism leading to lactic acid accumulation, metabolic acidosis and subsequent electrolyte imbalances. Accumulation of intracellular calcium and sodium occurs in addition to free radical formation, leading to cellular oedema, cell death and apoptosis [64]. When exposure to hypoxia is prolonged, the inflammatory response is more prominent, and the damage is more severe, hence pathological damage is more prominent [66,67]. Like hypothermia, hypoxia induces oxidative stress *via* ROS production, leading to damage in various body organs, among which, the heart and brain are the most sensitive [64,66]. Hypoxia is a stressor that produces biochemical and histopathological findings comparable to those produced by MH. Hypothermia induces pathophysiological changes that result in hypoxia to tissues [8,37,39], which might explain the degree of similarity between hypoxia and MH in the histopathology of damaged organs.

However, in hypoxia, the glycolytic pathway is primarily activated. Cells respond to hypoxia through expression of the hypoxia-inducible transcription factor (HIF-1) complex, which stimulates expression of multiple genes, including glucose transporters and genes mediating the glycolytic pathway. Hypoxia increases glucose uptake and stimulates the conversion of pyruvate into lactate [68]. This might explain the decreased serum glucose levels in the Hx group in the present study. On prolonged oxygen deprivation, HIF-1 decreases mitochondrial oxygen consumption and hence attenuates ROS in an attempt to enhance cell survival [68], which might explain the lesser organ damage and the lower oxidative stress compared with that of the SH group.

The stress hormones released under exposure to hypoxia induce lipolysis, and FFAs accumulate in the circulation. However, hypoxia also leads to decreased FFA uptake into cells and decreased FFA oxidation [69]. This explains the elevated FFA levels in the circulation and further explains the lack of lipids in the examined hypoxia-exposed organs in the present study.

## Conclusion

Cold exposure leads to various biochemical and histopathological changes. Biochemical changes include electrolyte disturbances and excess release of stress hormones, with consequent metabolic changes. Oxidative stress occurs in response to hypothermia and is aggravated by increased cold intensity. In our study, degenerative changes occurred in the brain, cardiac muscles, adrenal glands, liver, kidneys and skeletal muscle with lipid accumulation in the suprarenal glands and cells lining the renal medullary tubules. Although biochemical changes in response to hypothermia were also detected in response to hypoxia, they were less prominent under hypoxia and were comparable to those due to MH. Pathological changes detected under MH were also detected to some extent under hypoxia; however, no lipids accumulated inside the cells. Further clinical-level confirmatory studies are warranted.

The article "Histopathological, histochemical and biochemical postmortem changes in induced fatal hypothermia in rats" was published in 2021. Journal: Forensic Sci Res.

Human autopsy cases were excluded from the present study because of the nature of the weather in the authors’ country and the low number of hypothermia-induced fatalities. Furthermore, natural, and accidental deaths are not routinely subjected to autopsy in the authors’ country. No studies were performed with control groups subjected to other stressful conditions as the sources of trauma.

## Authors’ contributions

Mahrous Abdelbasset Ibrahim carried out the conception, design, the experiment, data analysis and drafted the manuscript. Sally Salem Mohammed carried out the histopathological investigations, data interpretation and helped to draft the manuscript. Hany G. Tammam participated in data analysis. Rehab Ibrahim Abdel-Karim participated in data analysis, interpretation and helped to draft the manuscript. Medhat Mohammed Farag carried out sample preparation and biochemical analysis. All authors contributed to the final text and approved it.
